# Design of Personalized Cervical Fixation Orthosis Based on 3D Printing Technology

**DOI:** 10.1155/2022/8243128

**Published:** 2022-04-30

**Authors:** Yangyang Xu, Xiangyu Li, Yafei Chang, Yi Wang, Lifang Che, Guopeng Shi, Xiaofen Niu, Haiyan Wang, Xiaohe Li, Yujie He, Baoqing Pei, Guoqiang Wei

**Affiliations:** ^1^Key Laboratory for Biomechanics and Mechanobiology of the Ministry of Education, School of Biological Science and Medical Engineering, Beihang University, Beijing, China; ^2^Department of Rehabilitation Medicine, Changzhi People's Hospital, Changzhi, Shanxi Province, China; ^3^Guilin Detachment of the Chinese People's Armed Police Force, Guilin Guangxi Zhuang Autonomous Region, China; ^4^Department of Rehabilitation Medicine, Ruyang County People's Hospital, Luoyang, Henan Province, China; ^5^Department of Anatomy, School of Basic Medical Sciences, Inner Mongolia Medical University, Hohhot, China

## Abstract

The movement of the cervical spine should be restricted throughout the rehabilitation phase after it has been injured. Cervical orthosis is commonly utilized in clinical settings to guarantee cervical spine stability. However, to date, the investigations are limited to patient-specific cervical fixation orthoses. This study provides a new idea for making personalized orthoses. The CT data of the patient's cervical spine were collected, then mimics were used for reconstructing the skin of the cervical spine, the Geomagic Studio was used for surface fitting, the Inspire Studio was used for structural topology optimization, redundant structures were removed, the resulting orthotics were postprocessed, and finally, it was printed with a 3D printer. No signs of pain or discomfort were observed during the wearing. The cervical spine range of motion in flexion, extension, lateral flexion, and rotation is all less than 8° after using the device. Low cost, quick manufacturing time, high precision, attractive appearance, lightweight structure, waterproof design, and practical customized orthotics for patients are all advantages of 3D printing technology in the field of orthopedics. Many possible benefits of using 3D printing to build new orthotics include unique design, stiffness, weight optimization, and improved biomechanical performance, comfort, and fit. Personalized orthotics may be designed and manufactured utilizing 3D printing technology.

## 1. Introduction

The most common causes of spinal trauma are severe traffic accidents, falls, and sports violence injuries [1, 2]. The current annual total rate of incidence is estimated to be 0.20-0.64‰ [3, 4]. Surgical treatment, intervertebral decompression, and spinal internal fixation are all required for severe traumatic spinal injuries. Patients are frequently needed to wear cervical fixation orthoses to ensure the effectiveness of internal fixation following surgery. Intervertebral segment fixation, local stability, preservation of a certain cervical spine posture, and injury stress prevention to protect the damaged site and enhance weight-bearing tolerance are all aims of cervical orthoses. Cervical orthoses are commonly used to treat a variety of clinical issues, including muscle spasms to extreme instability. The primary goal is to provide relief or support for the neck. The orthotics used in this research mostly help individuals with weak neck muscles. To increase their self-sufficiency and quality of life [5, 6], neck orthoses are mostly used to stabilize/fix the neck after trauma or surgery, to offer support for individuals with chronic neck pain, and to support weakening neck muscles [7]. The cervical fixation orthosis has been the standard of postoperative cervical fixation therapy since George Cottrell initially described and created it in 1964 [8]. Traditional neck orthotics are divided into three categories: A soft neck orthotics, which is mostly formed of foam rubber and coated with cotton wool, is the most basic; padded mandibular and occipital supports, as well as two or four stiff metal upright supports and shoulder supports, are the second kind; and the cervical thoracic orthosis falls into the third type, with a support comparable to column orthotics and a hard metal link between the front and back parts [9]. New orthotics must be developed to conform to the patient's body size and clinical consequences. To ensure suitable neck fixation, the new design idea should concurrently improve comfort, attractiveness, lightweight construction, and more steady contact pressure.

Plaster molds are used to create traditional orthotics. Low-temperature thermoplastic plates arise after the completed goods are large, require a long time to fabricate, and are costly [10, 11]; despite the fast manufacturing time, the orthoses are not attractive; they are thick and have major geometric flaws, as well as a lack of individualized comfort and function. Structures that are difficult to construct manually and have great accuracy can be designed using 3D printing technology [12, 13]. Traditional orthoses take roughly a week to make, but 3D printers may generate orthoses in just one day [14]. 3D printing technology, also known as additive manufacturing (AM), is a technique that can create new forms of orthotics that are individualized in terms of fit and shape [15]. 3D printing is a manufacturing technique that allows you to build complicated physical models and prototype components layer by layer straight from 3D computer-aided design (CAD) files, allowing you to create practically any complex solid three-dimensional design. Recent researches on personalized orthoses have focused on the upper and lower extremities, emphasizing the feasibility of AM in this area [16–18]. Few researches have considered this manufacturing procedure a realistic solution for the cervical area. The complicated role of cervical orthoses, which must support, prevent, or correct the spine, is to blame for this. Furthermore, therapeutic considerations must be balanced against other variables like comfort and aesthetic appeal. Long-term usage of cervical orthosis currently on the market is unpleasant, restricted, and poorly tolerated [19]. Devices that may be customized and configured individually for people with increasing neuromuscular neck weakness have been created [7]. Patients with amyotrophic lateral sclerosis can benefit from orthoses that give head support and improve their capacity to control head movement, according to research [20]. Hale et al. [21] demonstrated how to design and create cervical orthoses using a mix of 3D scanning and 3D printing technologies to give personalized services to patients.

Personalized medicine based on 3D printing technology is rapidly evolving at the moment, but there are few researches designs on cervical orthoses and a lack of clinical data, prompting researchers to recognize the need for further development and research of cervical orthoses. Orthoses must be customized according to individual needs to achieve the best performance results. Clinicians must keep in mind that the objective of a cervical orthosis is to support the head and neck while limiting cervical spine movement. The fundamental purpose of cervical spine support is to keep the neuroanatomical posture of the cervical spine safe. The cervical spine fixation orthosis developed in this study was designed to limit the movement of the cervical spine in any plane in terms of function, as well as to ensure the safety and stability of the cervical spine when it is severely unstable, to prevent the vertebra from impacting important nerve structures and causing irreversible nerve damage. It fits the characteristics of the patient's body surface to ensure that it is free from the compression load of the bone bulge of the head and neck, and the patient's experience should be comfortable; in terms of appearance, it is as beautiful as possible, and the hollow structure lessens the weight of the orthosis, improves the ventilation properties, and reduces the discomfort when wearing it in the summer, according to the principle. This study uses a mix of 3D scanning and 3D printing technologies to illustrate the development and deployment of a novel methodology for designing and constructing orthoses. This study demonstrates the development and application of a novel workflow for designing and fabricating orthoses, using a combination of 3D scanning and 3D printing technologies.

## 2. Materials and Methods

### 2.1. Research Object

In April 2021, a 53-year-old woman weighing 55 kg was hurt in a road collision. The posterior cervical single-door open-door laminoplasty, spinal nerve root exploration and release, and C3-C7 titanium plate internal fixation were all completed under general anesthesia. She was transported to the Department of Rehabilitation Medicine for rehabilitation treatment one week following the procedure. The CT data of the patient's cervical spine was collected, and the 128-slice spiral computed tomography (CT) machine (Siemens, Germany) scanner was used to scan the cervical; the scanning line was vertical to the body's central axis. The scanning parameters were as follows: slice thickness 1.25 mm, pitch 1.25 mm, thickness of reconstructed layer 0.625 mm, reconstruction pitch 0.625 mm, Fov30 × 30 cm, matrix 512 × 512 dpi, tube voltage 150 kV, and current 260 mA. This study was conducted in accordance with the Declaration of Helsinki. This study was conducted with approval from the Ethics Committee of Changzhi People's Hospital. Written informed consent was obtained from all participants' guardians.

### 2.2. Orthotics production plan

#### 2.2.1. Step A

Perform three-dimensional reconstruction of cervical spine skin, import the patient's cervical spine CT image in Dicom format into Mimics 21.0(Materialise, Belgium) software, select “Soft Tissue (CT)” in “Threshold”, add “Masks” to the skin, perform the “Caculate Part” operation.asks” to the skin, and perform the “Caculate Part” operation. A three-dimensional reconstructed cervical skin model was obtained.

#### 2.2.2. Step B

Import the 3D cervical spine skin model into the 3-matic 13.0 module in the “.stl” format, and select the rough outline of the orthosis through the “Lasso Aear Mark” function.

#### 2.2.3. Step C

The outline of the orthosis was imported into Geomagic Studio 2013 (Raindrop Geomagio Inc., USA) in “.stl” format, the model was processed, the noise was removed, spikes were removed, the surface was fitted, and a smooth surface was obtained.

#### 2.2.4. Step D

Altair Inspire Studio is an optimization simulation platform for designers. Its topology optimization tool, Inspire, is easy to operate, has a clear process and concise interface, and is easy to use. The orthosis surface is imported into Altair Inspire Studio 2018 (Atair Corporation. USA) in “.igs” format, and fixed constraints are imposed on the orthosis distal shoulder, back distal, and sternocleidomastoid midpoint position, on the upper edge of the orthosis that supports the head (including the chin, mandible, shoulder, scapula, and subclavian). The force generated by the weight of the head is 100 N; in order to make the model can resist more force, a load force of 200 N is selected [22]. Equidistantly apply multiple load forces perpendicular to the surface, all of which are 200 N, to simulate the effect of the force on the orthosis when the head is in motion. The material selection system comes with “ABS (Acrylonitrile Butadiene Styrene, elastic modulus: 200 Mpa, Poisson's ratio: 0.394.).” ABS is a thermoplastic polymer structure material with high strength, good toughness, and easy processing: select the entire orthosis surface as the design space; in the “Structure Simulation” menu, select “Topology Optimization”; target: maximize stiffness; mass target: 30% of the total volume of the design space; after the task is submitted, the software background automatically performs mesh division and finite element analysis and then determines the removal of elements in the design space according to the algorithm. The remaining units constitute the final topology scheme, so as to realize topology optimization and finally obtain the optimized model.

#### 2.2.5. Step E

After topology optimization, the model was imported into 3-matic 13.0 in “.igs” format, and “Wrap” was performed to increase the thickness, hollow out and modify the bony prominence, match with the patient's cervical spine model, adjust the size, and leave the installation space. Pad space, add buckles, and complete the model design of cervical orthosis.

#### 2.2.6. Step F

Adjust and display the CAD model.

#### 2.2.7. Step G

The cervical orthosis model was imported into Materialise Magics 21.0 in “.stl” format, and “model repair” was carried out; the parts were placed, the e-Stage module automatically added supports, and the printing platform and “.slc” file were exported. Import the print file into the 3D printer for orthosis printing (Figure 1).

### 2.3. Patient Wear and Evaluation

The adaptability and correctness of the constructed orthosis for patients are subjectively assessed. The orthosis is worn for 15-30 minutes, gradually increasing to 2 hours each time, and the comfort is measured using a chart questionnaire that considers 5 factors of satisfaction: appearance, weight, breathability, wearing operation, and material. The subjective feeling of comfort is divided into 7 grades (no discomfort, a little uncomfortable, very uncomfortable, extremely uncomfortable, a bit painful, very painful, and severe pain) [23], the satisfaction level is divided into 5 grades (very satisfied, satisfied, average, not very satisfied, and very dissatisfied), and the patient's skin condition is assessed (Figure 2). During sitting and standing exercises, the patient should wear orthotics. Adjust the time to the patient's comfort level. It should be worn at least 30 minutes at a time, with the time progressively increasing to 2 hours. Keep an eye on the patient's vital signs (blood pressure, pulse). If the patient felt any pain, the orthotics were taken off right away, and let the patient lie down and rest. Observe whether the wound is congested and purple, and ask the patient if there is a pinched region, if there is pain, and if there is a pinched area during the wearing process. When the orthosis is removed, the therapist looks for redness and swelling on the body surface. Three comfort level questionnaires were used to record the patients' subjective sensations. Fill out the comfort level questionnaire: the main purpose is for you to circle the region on the image below where you are uncomfortable and note your degree of discomfort on the chart (mark √ for 30 minutes; mark ○ for 1 hour; and mark △ for 2 hours).

## 3. Result

### 3.1. Cervical Fixation Orthosis Design Details

The cervical orthosis weighed 477 g, and it took 4 hours and 34 minutes to print. The substance is a durable and waterproof photosensitive resin. It has excellent skin wrapping and support. The overall hollow design has the advantages of lightness and ventilation; the cervical spine anterior opening design does not obstruct swallowing function and provides convenience for wound care and observation after the anterior cervical approach; the posterior cervical spine opening is designed to facilitate wound care and observation after the anterior cervical approach in accordance with the direction of cervical spine surgical opening; the supraclavicular area and inner side of the scapula are designed to limit the fixation effect of the cervical spine in all directions and ensure the postoperative effect of cervical interbody fusion (Figure 3).

### 3.2. Patient Questionnaire

The patient had no obvious discomfort during the wearing process and pointed out the position of the chin, and there was no obvious discomfort in other positions except for the pressure on the bilateral scapulae. The skin feels less supporting pressure, and the patient's wearing comfort increases when a sponge pad is put to the inside side of the orthotics. When a sponge pad is placed on the inside side of the orthosis, the skin feels less supported. After using the device, measure the patient's flexion at 5°, extension at 3°, left flexion at 5°, right flexion at 5°, and rotation at 7°, and joint range of motion in all directions is less than 8°, wearing orthoses for walking, sitting, and standing. (Figure 4). During the training, the patient's blood pressure is kept within normal limits, her pulse is 60-100 beats per minute, has regular breathing, and has no dizziness or vertigo symptoms, and she fills out a comfort level questionnaire (Figure 5). The results of the satisfaction questionnaire show that the patients are very satisfied with the appearance, weight, and breathability and are satisfied with the wearing operation and material.

## 4. Discussion

Orthotics were abandoned for a variety of reasons, including cost, size, difficulty in use, discomfort, and lack of customization. The majority of commercial collars are designed for acute use; however, long-term use of these collars is painful, restricting, and poorly accepted [19]. In this study, a personalized orthosis is a tailored design for the patient, such as the opening design of the wound or wounded area, which can be tuned for the biomechanical requirements of each portion to give improved functions, better match the curved surface, and improve aesthetics. 3D-printed orthotics have a number of advantages, including enough precision, a pleasing look, a lightweight structure, a waterproof design, sanitation, and ease of care.

This study presents an innovative and effective method for precisely adjusting and manufacturing orthotics with improved fit and custom functional characteristics. The hollow shape of the orthosis allows the clinician to see wounds and sutures in order to assess the healing process and situation; Baerg [24] and others have built a comparable structure. The hollow design efficiently avoids pressure sores because the projecting component of the bone increases the pressure on the skin, exceeding the skin's maximal capillary pressure and resulting in pressure sores. Hale et al. [21] employed 3D printing to create an orthosis for a patient whose cervical spine could not be erected owing to myelitis, and they got the same outcomes as this study, proving the superiority of this method. Sabyrov et al. [25] reported a novel design of a personalized neck orthosis made with fused deposition modeling technology, which reduced discomfort on the chin by constructing a unique structure, an expanded support section on the trapezius muscle. Comfort and stability were improved, and the excellence and application of 3D-printed novel cervical orthoses were proven, modeling of fused deposition. Prates [26] introduces a technique for creating a personalized 3D-printed multimaterial cervical orthosis for each patient that combines modern manufacturing technology with smart materials and biomimetic architectures to achieve a lightweight, waterproof, vented, sanitary, and comfortable fit. This novel approach and unique idea will be incorporated into the development of cervical orthosis products. Ambu et al. [27] describe the design, assessment, and production of a fused deposition model of a bespoke neck orthosis, and they want to improve the method by automating the steps of producing a CAD model for the use of AM neck orthoses in clinical trials of orthopedic therapies. There have been numerous studies comparing 3D-printed orthotics to traditional orthotics, with the conclusion that 3D-printed orthotics are more comfortable to wear [28–31]. Relevant research points out that with the effective use of CAD and 3D printing, smaller and lighter products can be obtained on medical products, reducing patient costs and benefiting patients [32]. CAD data may be saved for a long time; if an orthosis is destroyed or lost, it is simple to recreate the same product using the saved files; this is one of the advantages [33]. Compared with the existing research, the biggest advantage of this study is that the topology optimization method is used, which makes the orthosis look good in appearance, lighter in weight, and better in mechanical properties.

The findings of this study concentrated on changes in joint range of motion. Before the design began, it was decided if the cervical spine's range of motion in all directions needed to be entirely limited. There is room between the mandible and the location behind the occiput when the orthosis is worn. The goal is to make the cervical vertebra move somewhat, while also ensuring that it is not unstable and that there is some capacity for mobility. However, no report on how to manage these factors is currently available. It is beneficial to provide some space for mobility based on the patient's performance.

Various technologies for orthoses are constantly being developed. 3D printing is the most promising technology. The cost of 3D printing technology is also lowering due to the ongoing development and optimization of new materials [34]. As a result, all of these benefits are supporting the standardization of orthosis manufacture, resulting in improved treatment and outcomes [35]. With the advancement of printing material performance and printing technology, more study is required to establish the optimal printing technology and printing material for maximum applicability and durability. A customized cervical fixation orthosis was created and manufactured utilizing 3D printing technology as part of our study. The orthosis has a good fixation effect and is well received by the patients in terms of size, weight, convenience of use, and comfort. The process of orthosis creation, modification, printing, testing, and analysis allows design teams, particularly rehabilitation therapists, to generate new ideas, and the use of 3D printer technology opens the door to future revolutionary tailored goods [36]. In comparison to traditional methods, 3D-printed orthotics provide a high level of satisfaction and comfort. Choo [37] believes that 3D printing technology can replace traditional methods and is expected to be more popular in the future. The findings of this study concentrated on changes in joint range of motion. Before the design began, it was decided if the cervical spine's range of motion in all directions needed to be entirely limited. There is room between the mandible and the position behind the occiput when the orthosis is worn. The goal is to make the cervical vertebra move slightly and to ensure that the cervical vertebra does not become unstable. However, no report on how to control these factors is currently available. It is beneficial to leave some room for movement based on the patient's performance.

## 5. Conclusions

Personalized orthotic design and clinical effect studies were conducted through 3D printing technology combined with clinical cases, proving that the workflow of this study is feasible, is effective, and can bring benefits to patients. This study demonstrates the development and application of a novel workflow for creating cervical orthoses, using a combination of 3D scanning, topology optimized design, and additive manufacturing. It has been proven that the workflow of this study is possible and effective and may deliver advantages to patients using 3D printing technology mixed with clinical cases to undertake personalized orthotic design and clinical effect research. This study uses a mix of 3D scanning, topology optimized design, and additive manufacturing to illustrate the development and deployment of a unique workflow for constructing cervical orthoses. The next step in this study is to increase the number of patients by having a large number of patients wear neck orthoses, then follow up to get the patient's reaction to discomfort during use, as well as to assess the patient's cervical spine range of motion, provided support, flexibility in use, and appearance and comfort.

### 5.1. Strengths and Limitations of this Study

- This trial is a comparative effectiveness trial in a setting similar to the real-life clinical situation
- This article only shows a case of comfort assessment of cervical orthosis
- The evaluation results are subjective

## Figures and Tables

**Figure 1:** Schematic representation of design workflow and fabrication process of a custom orthosis. (a) Spiral CT scan. (b) 3D reconstruction of cervical skin. (c) This geometry is fitted. (d) Topology optimization of geometry. (e) Adjust the model structure and add a fixed buckle structure. (f) Schematic diagram of the CAD model. (g) This orthosis is obtained by 3D printing.

**Figure 2:** Patient questionnaire chart.

**Figure 3:** The design details of the cervical spine fixed orthosis.

**Figure 4:** Patient wears orthoses for walking, sitting, and standing.

**Figure 5:** Patient questionnaire chart feedback.

## Data Availability

The data used to support the findings of this study are included within the article. This is an article about the design of orthotics. The data is simple, and the range of motion of the cervical spine is obtained, including “After wearing, measure, the patient's flexion at 5°, extension at 3°, left flexion at 5°, right flexion at 5°, and rotation at 7°, and the range of joint range of motion in all directions is less than 8°.”
